# Blockchain-Based Information Supervision Model for Rice Supply Chains

This article has been retracted.

**DOI:** 10.1155/2022/2914571

**Published:** 2022-03-29

**Authors:** Jian Wang, Xin Zhang, Jiping Xu, Xiaoyi Wang, Haisheng Li, Zhiyao Zhao, Jianlei Kong

**Affiliations:** ^1^School of Artificial Intelligence, Beijing Technology and Business University, Beijing 100048, China; ^2^Beijing Key Laboratory of Big Data Technology for Food Safety, Beijing Technology and Business University, Beijing 100048, China; ^3^School of Computer Science and Engineering, Beijing Technology and Business University, Beijing 100048, China

## Abstract

Rice is a major food crop around the world, and its various quality and safety problems are closely related to human health. As an important area of food safety research, the rice supply chain has attracted increasing attention. Based on blockchain technology, this study investigated problems of data privacy and circulation efficiency caused by complex rice supply networks, long circulation cycles, and various risk factors in each link. First, we deconstructed the quality and safety of each link of the rice supply chain at the information level and established a key information classification table for each link. On that basis, we built a rice supply chain information supervision model based on blockchain. Various encryption algorithms are used to secure the sensitive data of enterprises in the supply chain to meet regulators' needs for efficient supervision. Moreover, we propose a practical Byzantine fault-tolerant consensus algorithm that scores the credit of enterprise nodes, optimizes the selection strategy of master nodes, and ensures high efficiency and low cost. Then, we built a prototype system based on the open-source framework of hyperledger fabric, analyzed the model's viability, and implemented the system using cases. The results indicated that the proposed system can optimize the information supervision process of rice supply chain regulators and provide a feasible solution for the quality and safety supervision of grain and oil.

## 1. Introduction

In recent years, consumers have paid increasing attention to food quality and safety, which provide a basic guarantee for human health and are directly related to improving people's lives [1]. Rice is among the world's major food crops, but in recent years, various quality and safety problems have arisen, such as cadmium-laced rice, mercury-laced rice, and aging grain [2–4]. Such problems can not only affect human health but also threaten social stability. It is necessary, therefore, to establish a safe and efficient rice supply chain information supervision system. Compared with other foods, rice is characterized by long supply chains, complex supply networks, long circulation cycles, and numerous risk factors in all links [5, 6]. Moreover, each link of the rice supply chain is relatively independent, and there is little information exchange between them. It can be difficult, then, for enterprise nodes in the supply chain to trust each other, and supervision efficiency is low [7, 8]. In addition, traditional supervision systems rely on a centralized database to store data. This can give rise to problems such as enterprises tampering with detection data in different links of the supply chain, which compromises the credibility of supervision results [9, 10].

Blockchain technology can provide effective solutions for issues related to centralization, security, and tamperability [11–13]. Blockchain can automatically execute a code according to business rules set by the system and can record the whole process in the chain to reliably transfer information, logistics, and capital flow information in a supply chain [14, 15]. In recent years, researchers have investigated the supervision and management of blockchains combined with food and agricultural product supply chains. They have focused on areas such as establishing product identification through various technologies and developing supply chain management systems for data uploading, real-time monitoring, early risk warning, and information tracing using sensor technologies [16–19]. It has been found that blockchain can improve data security and traceability for food-related supply chains and provide a guarantee for food quality and safety. However, there is still much room for improvement in the areas of blockchain storage modes, consensus overhead, and rice supply chain information supervision.

In light of the above, this study deconstructed and analyzed the quality and safety information of each link of the rice supply chain at the information level and established a key information classification table for each link. Then, a rice supply chain information supervision model was constructed based on blockchain. The model adopts a hierarchical privacy encryption and storage mode, as well as a practical Byzantine fault-tolerant consensus algorithm based on credit scoring (CPBFT). Finally, a prototype system was designed, and the model and system were analyzed to provide a reference for the current theoretical research and actual construction of rice supply chain information supervision system.

## 2. Related Work

Researchers have investigated the application of blockchain technology in related fields from different perspectives. Baralla et al. [20], for example, developed a blockchain-based system to manage and trace the food supply chain, using smart contracts to ensure the credibility of the whole process. Based on an analysis of the wheat-processing supply chain, Zhang et al. [21] proposed a blockchain-based grain and oil supply chain system architecture using a multimode storage mechanism. Wang et al. [22] proposed a framework based on consensus and smart contracts to achieve traceability and sharing in the agricultural product supply chain and improve the integrity and security of transaction records. In their model, data are stored in an interstellar file system, and the data hash is stored in the blockchain network, which saves storage space and ensures security. Mao et al. [23–25] built a blockchain-based food supply chain trading system to provide more reliable and authentic information. Pigini and Conti [26] used Near Field Communication (NFC) technology to achieve effective traceability and safety tracking to collect product information in all links of the food supply chain. Salah et al. [27] analyzed the traceability and business processes of the soybean supply chain and proposed using smart contracts to control and ensure the safety and credibility of supply chain information.

The aforementioned studies addressed the security problems of food supply chains to a certain extent. However, with the rapid expansion of supply chain nodes, existing traditional consensus modes have too much overhead, and sharp increases in the amount of data have corresponding requirements for consensus security. Researchers have sought to solve this problem by improving the blockchain consensus algorithm. Liu et al. [28], for example, improved the Delegated Proof of Stake (DPOS) consensus algorithm to keep the consensus process from being controlled by a few nodes. Meanwhile, to achieve node consensus in large-scale distributed systems, Li et al. [29] proposed an extensible multilayer PBFT consensus mechanism that groups nodes hierarchically and limits communication within the group, such that PBFT consensus is not limited to small consensus networks. In rice supply chains, however, the key data in each link are complex, and enterprise entities cannot form a unified standard. It is necessary, then, to adopt a targeted consensus scheme, that is, to reduce the consensus cost and ensure consensus reliability at the same time. In addition, because the nodes in the blockchain are not completely anonymous, there are privacy risks, which necessitate privacy encryption for uplink data.

To meet these challenges, this study analyzed the information for each link in the rice supply chain and output a classification table of key information for each link. Combining the principles of cryptography and blockchain, we proposed a data encryption and storage mode that protects the sensitive data of supply chain enterprises and meets the needs of regulators for efficient supervision. In addition, our proposed credit score-based PBFT consensus algorithm reduces the probability that the master node is a Byzantine node and ensures high efficiency and low overhead. In summary, this research can help optimize regulators' information supervision processes in rice supply chains and provide a feasible solution for rice quality and safety supervision in the future.

## 3. Analysis of Supply Chain Process and Key Information

Many enterprises are involved in each link of the rice supply chain, including growers, purchasers, storage enterprises, processing enterprises, logistics enterprises, and distributors. The rice supply chain is therefore characterized by a long life cycle and complex links. From rice planting to sales, there are many potential safety hazards in the supply chain, which are summarized in the following:

1. In the planting process, rice needs to absorb a large amount of water, which makes it more vulnerable to pollution than other crops. Farmers' fertilization practices are not always standardized. Some even irrigate farmland using untreated domestic sewage and industrial wastewater, resulting in excessive heavy metal pollution [30].
2. Rice processing is a lengthy process, and problems such as broken rice and fumigant residue easily arise in the process of impurity removal [31]. China's rice-quality standards stipulate that no flavor or pigment is allowed in rice. Yet, to increase profits, some enterprises in China add fragrance to rice or treat it to increase its brightness. When polishing rice, it not only adds water but also illegally adds mineral oils, thus processing ordinary rice into “poisonous rice.”
3. With regard to packaging, the plastic woven bags mainly used for rice commodities offer a simple, low-price packaging method. However, the material has a poor moisture barrier and moisture resistance, resulting in problems such as oxidization and mildew.
4. Storage and transportation links: improper warehouse storage makes rice prone to mildew. In addition to changing the color of rice, mildew can produce harmful molds and microorganisms [32].
5. The sales link of rice is widely distributed and contains a large amount of information. As the terminal link of the supply chain, it directly faces consumers. If there is an information supervision problem in this link, it can seriously affect the whole supply chain.

In summary, the types of hazards in each link of the rice supply chain are complex, and safe and efficient supervision is needed. However, traditional blockchain supervision systems generally have problems such as large differences in inspection standards and inconsistent data storage formats in all links of the supply chain. It is difficult to effectively enter the multilink information of a complex supply chain. It is also difficult to build models and systems based on these data in the follow-up process, making it difficult to solve the problem of rice quality in terms of data security.

Based on the rice supply chain process and the business characteristics of enterprises in the supply chain, we divided the rice supply chain into 13 links and five types of key data: main information, basic information, environmental information, hazard information, and transaction and price information (Table 1).

The subject information is the enterprise information in different links of the supply chain, including the enterprise name, the person in charge, and contact information. The basic information is the information recorded by the enterprise staff in each link, such as rice type, sampling inspection record, rice milling method, and whether it is genetically modified. Environmental monitoring information is the information recorded by sensors in the supply chain, including temperature and humidity, carbon dioxide concentration, and real-time photos. Hazard information mainly refers to the content of mycotoxins, pesticide residues, and heavy metals in rice during sampling inspection. Mycotoxins mainly include aflatoxin B1, ochratoxin A, and deoxynivalenol. Heavy metals include lead (Pb), cadmium (Cd), Mercury (Hg), arsenic (As), and chromium (Cr). Pesticide residues include chlorpyrifos, triazophos, carbofuran, and bensulfuron methyl. Transaction records and price information include the commercial information circulating among various links, and their confidentiality is high. Table 1 summarizes the key information in each link. Taking the processing link as an example, processing enterprises accept rice stored in multiple granaries, including storage enterprises. After the rice is transported to the processing plant, the processing plant also needs to carry out various processes, such as removing the husk, rice milling, color selection, and polishing. This study regarded the abovementioned processes as independent links. Detailed information classification can further optimize the process architecture of the supply chain business system and can be used as the basis for establishing an information supervision model for the safety and quality of the rice supply chain.

## 4. Blockchain-Based Supervision Model for Rice Supply Chain Information

Traditional rice supervision systems store supply chain information in a central database. Its supervision timeliness is poor, data are easily tampered with, flow between enterprises is difficult, and the enterprise data query efficiency is low. A blockchain stores enterprise data with a distributed ledger instead of a central database to achieve data sharing and value transfer between upstream and downstream enterprises in a supply chain. Using blockchain technology, an improved consensus algorithm, and the principle of cryptography, this study built a rice supply chain information supervision model based on supply chain processes and the characteristics of enterprises in the chain. The model includes not only complete supervision of the supply chain but also government agency supervision, as well as the data uploading and data sharing of enterprises. Querying and consumer commodity traceability are employed to achieve integrated supervision. In this way, rice information can be supervised and managed from the supply chain, which ensures the security and authenticity of data circulated in the supply chain. Meanwhile, it reduces the information gap between consumers, regulators, and enterprises in the supply chain and avoids the generation of information islands.

This study regarded each link in the rice supply chain as a node in the blockchain, and each node corresponds to a cloud database. Each node in the supply chain invokes a smart contract deployed in the blockchain network through the supervision system and carries out network consensus through an improved PBFT consensus algorithm. Enterprises in all links can encrypt and store the data in the system through this system. After blockchain network consensus, plaintext and ciphertext data in the supervision system are recorded in a cloud database, and a small part of the plaintext data, information summary, and key are saved in the blockchain network (Figure 1).

Combining regulatory authorities and supply chain enterprises and based on the key information classification table, we standardized the data uploading or traceability of supply chain links (e.g., production, processing, warehousing, transportation, and sales), which can achieve effective information supervision of the entire rice supply chain.

The model mainly includes rice supply chain network nodes, data hierarchical encryption, storage mode, and CPBFT. The data hierarchical encryption and storage mode combined symmetric encryption and hash encryption algorithms to ensure the security and privacy of the data uploaded to the blockchain network and the cloud database in the process of circulation and storage. Advanced Encryption Standard (AES) is used to ensure data confidentiality. It is characterized by that both sides of communication use the same key in the process of encryption and decryption. Hash encryption algorithms can compress arbitrary length data into information summary of fixed length to realize digital signature and data integrity. As a partial synchronous pattern consensus algorithm, PBFT has been widely used in the alliance chain. The algorithm can solve the Byzantine problem, which is relatively efficient and widely used [33]. However, when the algorithm is applied to the supervision of agricultural products with many coverage links, there are still some problems, such as high overhead, low throughput, and low performance. CPBFT introduces the credit-scoring mechanism in PBFT, which scores and grades the credit of supply chain enterprise nodes to ensure the efficiency of consensus. At the same time, the algorithm improves the reliability of supply chain supervision. In addition, based on the model, this study designs the information supervision prototype system, constructs the system infrastructure, and analyzes the complete operation process of the system.

### 4.1. Hierarchical Data Encryption and Storage Mode

Based on the above classification of key information in each link of the rice supply chain, as well as the integration of data privacy, encryption algorithm security, algorithm time complexity, and space complexity in each link, we performed the hierarchical encryption and secure storage of supply chain circulation data.  Figure 2 shows the data flow in the encryption and storage mode.

We mainly used the AES encryption algorithm and SM3 password hash algorithm to encrypt and decrypt the supply chain information. The AES encryption algorithm uses ECB and CBC working modes. The difference between AES working modes is reflected in the association between plaintext data blocks, although the processing flow inside the AES encryptor is the same. Algorithm 1 shows the AES encryption process, and Algorithm 2 shows the decryption process. NR is the number of encrypted rounds. For different key lengths, the number of rounds is different, and W is the extended key array. The SM3 hash algorithm is a commercial hash algorithm standard published by the State Encryption Administration of China. The algorithm has excellent anticollision ability and is very suitable for privacy data encryption in a rice supply chain. For a plaintext message *m* with a length of less than 264 bits, the SM3 hash algorithm generates a hash value (ciphertext) after filling and iterative compression. The hash value length is 256 bits. Algorithm 3 shows the encryption process.

#### 4.1.1. Level I Privacy Data Encryption

Hazard information is defined as level I privacy data. In this mode, the AES algorithm ECB mode is used to encrypt level I privacy data and then transmit it to the cloud database. In this mode, the encryption of each plaintext block is completely independent. The data are grouped with 128 bits, and the remaining insufficient bits are filled to reach the integer multiple of the packet:

(1) $$\begin{array}{c} x_{1},x_{2},x_{3}\ldots . \end{array}$$

Each group of data and the key of the same length are used as input, and new data packets are generated by independent encryption. The same is true for decryption. The encryption process is

(2) $$\begin{array}{c} y_{1}=E_{k}\left(x_{1}\right),y_{2}=E_{k}\left(x_{2}\right),y_{3}=E_{k}\left(x_{3}\right)\ldots . \end{array}$$

The decryption process is

(3) $$\begin{array}{c} x_{1}=D_{k}\left(y_{1}\right),x_{2}=D_{k}\left(y_{2}\right),x_{3}=D_{k}\left(y_{3}\right)\ldots . \end{array}$$

The AES algorithm ECB working mode can carry out a large number of parallel calculations, which is suitable for rice hazard information with large amounts of data. In this mode, the data key is randomly generated by the algorithm and uploaded to the blockchain network for storage to ensure the randomness and security of the key and mitigate the risk of key disclosure in symmetric encryption.

#### 4.1.2. Level II Privacy Data Encryption

Transaction records and price information are defined as level II private data. For level II private data, the AES algorithm CBC mode is used for encryption, and ciphertext data are transmitted to the cloud database.

In the process of privacy data encryption, the first plaintext data packet is XOR with the randomly generated initial vector IV. Then, packet encryption is carried out, and the ciphertext output by this group and the XOR of the next plaintext packet are used as the input of the next packet encryption. In this way, until encryption is completed, the decryption process is the same.

Encryption process:

(4) $$\begin{array}{c} y_{0}=IV,\\ y_{1}=E_{k}\left({\text{y}}_{0}⊕x_{1}\right),\\ y_{2}=E_{k}\left({\text{y}}_{1}⊕x_{2}\right)\ldots . \end{array}$$

Decryption process:

(5) $$\begin{array}{c} y_{0}=IV,\\ x_{1}=D_{k}\left(y_{1}\right)⊕y_{0},\\ x_{2}=D_{k}\left(y_{2}\right)⊕y_{1}.... \end{array}$$

The output of each ciphertext in this mode is related to its corresponding plaintext packet and all previous plaintext packets; thus, the ciphertext generated by the same plaintext may be different. Therefore, compared with the ECB mode, the CBC mode has stronger security and is suitable for commodity value guarantee with a higher security level. In addition, in this process, the data key is generated and stored in the same way as with level I privacy data.

#### 4.1.3. Level III Privacy Data Encryption

Subject information, basic information, and environmental information are defined as class III privacy data. For subject information, the amount of data is small, and the degree of importance is high. This mode adopts the method of directly transmitting data to the blockchain network. For all level III privacy data, the SM3 cryptographic hash algorithm is used for encryption. The algorithm first fills the data and then expands the filled data, iteratively compresses the expanded data, and finally generates an information summary with a length of 256 bits. Finally, the encrypted information summary is uploaded to the blockchain network, and the level III privacy data are uploaded to the cloud database in plaintext. The compression function of the SM3 cryptographic hash algorithm has a similar structure to that of SHA-256, but the structure of the compression function of the SM3 cryptographic hash algorithm and the design of the message expansion process are more complex. Each round of the compression function uses two message words, and each round of the message expansion process uses five message words, which can further ensure that high-privacy data are nontamperable.

### 4.2. Practical Byzantine Fault-Tolerant Consensus Algorithm Based on Credit Score

The PBFT algorithm is a partially synchronous mode consensus algorithm. To ensure that nonfault nodes execute client requests in the same order, third-order broadcast communication is needed to ensure security in the asynchronous mode, resulting in a great deal of communication overhead. At the same time, PBFT lacks the mechanism of troubleshooting nodes, and the selection of master nodes is arbitrary. The probability of selecting Byzantine nodes as master nodes is high, and the frequent replacement of master nodes greatly affects system efficiency [28, 34]. Therefore, this study improved the original PBFT algorithm and designed CPBFT (PBFT based on credit score) according to the characteristics of rice supply chains. Taking the transaction time and honesty of the nodes in the rice supply chain as the main reference factors, we scored the behavior of all nodes participating in consensus in the supply chain. The credit-scoring model divides the nodes into fault, ordinary, supervision, and candidate nodes according to the score and then optimizes the selection strategy of the main node, reduces the possibility of the main node becoming a Byzantine node, reduces the amount of view switching, and improves the efficiency of the information supervision system.  Figure 3 shows the classification and conversion mode of consensus nodes.

#### 4.2.1. Credit-Scoring Mechanism of Nodes

In this model, it is necessary to first conduct multiple rounds of PBFT consensus and then select the consensus set, eliminate nodes that fail in the consensus process or send messages inconsistent with most nodes, and conduct node credit scoring to remove most nonsystem interference factors.

After each correct consensus, the credit score of the corresponding node is added *β*. After *n* rounds of consensus, all honest nodes will correctly complete the consensus, and the node's credit score will be *η*. The traditional PBFT consensus algorithm has 3*f* + 1 nodes, and at least 2*f* + 1 honest nodes can complete consensus. If a malicious node wants to join the consensus set, it must be honest every time. At this time, the credit score of more than 2*f* + 1 nodes will be divided into *η* and is marked as an honest node. This will be reached within specified time *η*. The node with the score is marked as an ordinary node and can only participate in consensus. A node that fails to reach the score is regarded as a fault node. After multiple consensuses, according to the credit score of the node, the nodes participating in consensus can be divided into ordinary, supervision, candidate, and fault nodes. These nodes perform different functions in the consensus to maintain the stable operation of the rice supply chain information supervision system.  Table 2 shows the specific node division method.

In the unimproved PBFT consensus mechanism, the master nodes are randomly selected by formula *p*=*v*mod|*R*|, where *p* is the master node number, *v* is the view number, and |*R*| is the number of nodes. The probability that the selected master node is a Byzantine node is 1/3. In this model, the node with the highest score among the candidate nodes is selected as the master node of the next view. If there is no single node with the highest score, the system randomly selects a node with the highest score among the candidate nodes as the master node. After a period of time *t*, the master node resets the node credit score and downgrades to an ordinary node to avoid the problem of overcentralization of the system. The main node selection mechanism of this model reduces the possibility of a Byzantine node becoming the main node, reduces the number of attempts to switch, reduces communication overhead, and improves system efficiency and security.

In the process of consensus, there are often objective fault nodes and subjective malicious nodes caused by unavoidable physical conditions, such as enterprise host failure, communication system delay, and supply chain link change. The role of the monitoring node is to eliminate the problem nodes in these situations. In the process of consensus, the monitoring node can record information that has been judged malicious by the system and then deprive it of consensus authority. In addition, the monitoring node can also record the node that does not send feedback information to the client within the specified time, or the feedback information is inconsistent with the feedback information of most nodes. Then, the system will mark the node as a failed node and temporarily deprive it of consensus authority. When the problems of malicious or failed nodes are repaired, the system will initialize them as ordinary nodes. The existence of a supervision node further reduces the possibility of fault nodes in the consensus node, improves consensus efficiency, and reduces system overhead.

#### 4.2.2. Consensus Process

Figure 4 shows the CPBFT algorithm flow. After a consensus is started, all nodes are initialized and classified according to their credit scores. However, since the credit scores of the nodes are all 0, all nodes are ordinary nodes at the beginning, and the primary node is randomly selected according to the *p*=*v*mod|*R*| formula for consensus. After multiple consensuses, each node receives a corresponding credit score, and the node credit score system is gradually established. The model divides all nodes into four types with different functions and permissions and selects the main node according to the node credit-scoring mechanism. After the client sends the request, the master node broadcasts the proposal. If the replica node does not respond, the mechanism determines that the master node has a problem and records the delayed response information to the monitoring node. Then, the monitoring node judges whether the primary node is a failed node or a malicious node. Then, the mechanism will perform credit score reduction and node consensus authority deprivation for the corresponding nodes. The consensus process then returns to the node classification stage after view switching and finally reclassifies the nodes to select a new primary node for consensus. If the master node is an honest node, the consensus is completed at one time, and the algorithm will add points to the node that successfully records the information to the local node.

### 4.3. Design of the Information Supervision Prototype System

Based on the above model and the needs of all links in the rice supply chain, we designed a rice supply chain information supervision prototype system.  Figure 5 shows the system architecture, which is divided into application layer, consensus layer, storage layer, and perception layer.

As the data-acquisition end of the system, the sensing layer mainly collects the various business data and hazard information of supply chain enterprises through temperature and humidity sensors and infrared scanning and photographing equipment. It then transmits the data to the data storage layer through wireless sensor networks, 4G/5G, Wi-Fi, and other networks. The storage layer includes a cloud database and hyperledger fabric blockchain platform storage, in which data in the blockchain are stored in the form of files. Enterprises first perform data cleaning, transformation, and fusion and then encrypt and store data according to its privacy level through smart contracts. The hierarchical encryption and storage mode can ensure storage efficiency, decentralize data, and make data more secure and reliable. Meanwhile, this mode also facilitates user data query. The consensus layer encapsulates the improved consensus algorithm and mechanism. The credit-scoring model divides the consensus nodes into four categories, which can enable highly decentralized nodes to efficiently reach consensus on the effectiveness of block data in a decentralized blockchain network. The application layer provides corresponding functions to regulatory authorities, enterprises, and consumer users in the form of web pages and mobile apps. Further, it divides authority levels according to different users, mainly including information traceability, enterprise authority management, and supply chain supervision functions. It can also observe the number of nodes and score changes in real time.

The system adopts a hyperledger fabric open-source blockchain platform to construct the supply chain blockchain network. Its essence is the uploading and querying of the blockchain ledger and cloud database by supply chain node users through the client interface. The system adopts a B/S structure, CentOS 7 as the operating system; Docker 18.09 as the container engine; and go, JavaScript, HTML, and CSS for program development. CouchDB, LevelDB, and MySQL are used as database servers. MySQL is the main data storage database, and CouchDB and LevelDB are the status databases in the blockchain network. The state database is just an index view in the transaction log in the chain and can be regenerated from the chain at any time. Before data transactions, the state database will be automatically restored when the peer node starts or is generated as needed. LevelDB stores chaincode data as key value pairs, while CouchDB, which is mainly used in this system, uses JSON to store data, which can support richer queries.

In this study, different users who log in to the system have different permissions, which can be achieved by the hyperledger fabric's own management user ID and membership authentication function for all blockchain participants. Moreover, the fabric access control list can also enable different users to authorize different permissions.  Figure 6 shows the system sequence diagram. The personnel of multiple production, processing, transportation, packaging, and sales enterprises and regulatory agencies in the supply chain can use the system, and the user has the authority to upload and query data. Users log in to the system and upload data. At this time, the system calls up the smart contract and encrypts it according to the data privacy level of the rice supply chain. The encryption key is randomly generated by the system. Part of the data is saved to the traditional database, and the other part of the data and the key participate in node consensus and upload to the blockchain. At the same time, the system updates the enterprise node credit score of the supply chain to ensure efficiency consensus.

## 5. Performance and Effect Analysis

### 5.1. Model Analysis

In the practical application of a traditional rice supervision model, due to the use of a central database, data are easily tampered with, and enterprise data traceability and query efficiency are low. Blockchain stores enterprise data with a distributed ledger instead of a central database, which can achieve data sharing and value transfer between upstream and downstream enterprises in the supply chain. Based on rice supply chain processes and the business logic of enterprises in the chain, we built an information supervision model using blockchain, an improved consensus algorithm, and cryptography principles to ensure the safe, efficient flow of data in the chain.

In our model, symmetric and hash encryption algorithms are used to encrypt rice supply chain data twice before data connection. The blockchain network stores a small amount of plaintext data, information summary, and keys at a high security level. Most ciphertext and plaintext data are stored in a cloud database, which can ensure the security of information storage and circulation in the whole system. In addition, this mode differentially encrypts different data safely registered in the supply chain information flow, standardizes the data storage and management process of the whole system, completes the hierarchical storage of data, and makes system resource investment proportional to data importance. In this mode, various encryption algorithms are used to ensure the confidentiality, integrity, and availability of sensitive data. This helps protect the key sensitive data of rice supply chain enterprises; the hierarchical structure can also meet the needs of regulators for efficient supervision.

In terms of the safety of the algorithm, the selection of master node is arbitrary in the consensus process of PBFT. The algorithm can select the master node in turn according to the node number. CPBFT uses PBFT as the consensus core, and its intragroup consensus and global consensus antiattack capabilities are consistent with PBFT. The following focuses on the security performance of CPBFT against witch attack and conspiracy attack.

Sybil Attack refers to Byzantine node illegally inventing multiple identities to attack the network. In this study, the credit-scoring method is used to elect high credit nodes to participate in the consensus, while the nodes with low credit will be stripped of the authority of consensus by the system so as to reduce the probability of Sybil Attack.

Collusion attack means that multiple Byzantine nodes give a trust evaluation higher or lower than the actual level, which makes the trust value of the evaluated node deviate from the actual trust value. When the total number of Byzantine nodes in CPBFT does not exceed 1/3 of the total number, even if all Byzantine nodes collude, the system can still reach a correct consensus. And once malicious behavior occurs in the consensus proposal, the node is highly likely to be determined as a Byzantine node, and the monitoring node can record the information that has been determined as a Byzantine node by the system and then deprive its authority of consensus. Therefore, the node collusion attack can only increase the opportunity for Byzantine nodes to enter the set of alternative nodes through voting collusion, and the node credit-scoring mechanism of CPBFT can adjust and divide the credit score in real time according to the situation. When there are great differences in the credit evaluation of the attacked node, the system will change the parameters in the mode of division in Table 2 in real time to reduce the impact of collusion attack on consensus security so as to ensure the high reliability of the candidate node.

In addition, we conducted a system simulation on a hyperledger fabric platform and compared the traditional PBFT algorithm with the proposed CPBFT algorithm in terms of total communication between nodes and throughput. The communication overhead of the node was directly proportional to the number of communications between nodes in the consensus process. The main purpose of the CPBFT algorithm is to reduce the number of failed nodes in the consensus node to reduce communication. In the system simulation, one-third of the nodes were set as fault nodes. As shown in Figure 7, the communication of the CPBFT algorithm increases slowly, while the communication of the PBFT algorithm before improvement increases rapidly. Therefore, it can be seen that the CPBFT algorithm can effectively reduce communication overhead and broadband pressure.

Throughput refers to the number of transactions completed in a unit of time. CPBFT can effectively reduce the number of consensus nodes and shorten communication time. The probability that the master node is a reliable node is higher, the probability of error is smaller, the amount of view switching is reduced, and the time to complete consensus is shortened. For our experiment, we sent 800 requests to the client, recorded the number of transactions that could complete consensus per second, and tested it with different numbers of nodes.  Figure 8 shows the CPBFT algorithm. With the increase in the number of nodes in the network, the throughput of both algorithms shows a downward trend. Overall, however, the throughput of the CPBFT algorithm is much higher than that of the improved algorithm.

### 5.2. Systematic Analysis

After the field investigation of several rice enterprises, we initially chose to apply the system to a grain and oil enterprise in Changde City, Hunan Province, China, to verify the system's effectiveness. The enterprise's industry involves all links of the rice supply chain. All links have complete monitoring and inspection equipment and stable communication, and all data records are detailed and complete. However, as a result of internal information storage among enterprises and various exchanges between companies, the difficulty of supervision is further increased. In addition, all supply chain data of the enterprise are stored in the central database, and data security is difficult to ensure. Therefore, the proposed rice supply chain supervision system was selected to optimize the supervision and management ability of the enterprise.

Figure 9 shows the system interface.  Figure 9(a) is the login interface of the supervision system. After logging in to the system, a supervisor user with administrator authority can supervise and manage all circulating data in the rice supply chain. After logging in to the system, the enterprise user can upload and query information for the entire rice supply chain. The supervision user can search and query all data uploaded by an enterprise in the supply chain supervision interface, including its main information, basic information, hazard information, environmental information, and transaction and price information. As shown in Figure 9(b), all query information is the main data of the supply chain enterprise, which is encrypted and uploaded to the blockchain network and cloud database by the system. The system decrypts the plaintext data again. This mode effectively ensures security and privacy in the process of data storage and transmission. If it is verified as bad data, the regulator can mark the data and conduct a secondary sampling inspection of the information to finally determine whether the enterprise information is true and reliable and whether the rice quality is good. Users can query the information and stored data of each block in the privacy data management interface of the enterprise. Moreover, the user can decrypt the stored data according to the privacy level, as shown in Figure 9(c).  Figure 9(d) shows system consensus management. The main interface is a visual interface. The user can see real-time changes in the total number of consensus nodes and real-time changes in the type proportion of consensus nodes. Users can also select an enterprise node to view real-time changes in the credit scores of the node. Regulators can learn the latest change trend in consensus nodes through the consensus management function and adjust the credit score value in a timely way to improve consensus efficiency.

Compared with traditional systems, the proposed rice information supervision system has a detailed division of permissions. Regulators can query all supply chain circulation data in the system, while enterprise users can upload data and view node consensus. The corresponding permissions are different according to the different supply chain links of the enterprise. In addition, the regulator can query information and analyze privacy in real time according to data privacy level to determine the authenticity of enterprise information and the security of rice-quality data. Moreover, while monitoring the supply chain nodes, the system's visual interface can more intuitively show the data transmission efficiency of the supply chain.

## 6. Conclusions

The traceability, decentralized, and tamper-resistant characteristics of blockchain technology are in line with the requirements of information supervision system, and blockchain technology has broad development prospects in the field of information supervision system for rice supply chains. This study deconstructs and analyzes the quality and safety information of each link of the rice supply chain at the information level and establishes a key information classification table for each link. Combining cryptography with the characteristics of rice supply chains, a hierarchical data encryption and storage mode is proposed to ensure the security and privacy of data uploaded to the blockchain and cloud database in the process of circulation and storage. In addition, a scoring mechanism is introduced into the consensus process of the blockchain network. Supply chain enterprise nodes are scored to improve consensus efficiency. The improved consensus algorithm also improves the reliability of supply chain supervision.

Verified using practical cases, this research can help optimize regulator information supervision processes in rice supply chains, and the proposed rice supply chain information supervision system can provide a feasible solution for grain and oil supervision. The proposed approaches in the paper can combine other deep-learning algorithms to study the identification and prediction problems, and can be applied to other fields such as signal processing and engineering application systems [35–41].

## Figures and Tables

**Figure 1:** Rice supply chain information supervision model.

**Figure 2:** Hierarchical data encryption and storage mode.

**Figure 3:** Category and transformation of consensus nodes.

**Figure 4:** The process of CPBFT.

**Figure 5:** The information supervision prototype system architecture.

**Figure 6:** Sequence diagram of the information supervision prototype system.

**Figure 7:** Comparison of communication.

**Figure 8:** Comparison of throughput.

**Figure 9:** Front-end interface of the prototype system. (a) Supervision system login interface. (b) Supply chain supervision interface. (c) Privacy data management interface. (d) System consensus management interface.

**Algorithm 1:** Process of AES encryption.

**Algorithm 2:** Process of AES decryption.

**Algorithm 3:** Process of SM3 encryption.

**Table 1:** Key data of each link in the rice supply chain.

Links in rice supply chain		Key data classifications				
		Main information	Basic information	Environmental information	Hazard information	Transaction and price information
Plant		Identity information of growers; planting license information; contact information; business license information (optional)	Seed source; rice varieties; origin information; planting and harvesting time; pesticide and fertilizer information and use records	Pictures of rice growth cycles; real-time ambient temperature; real-time ambient humidity; actual illumination intensity of environment; soil moisture content	Pictures of rice growth cycles; real-time ambient temperature; real-time ambient humidity; actual illumination intensity of environment; soil moisture content	Seed price; fertilizer price; total cost; selling price; collect and store enterprise information
Acquisition and storage	Acquisition	Enterprise name; business address; corporate information; person in charge of relevant links; license information; enterprise contact information	Pesticide sampling inspection records; transgenic or not	None	Mycotoxin: fumigant and insecticide residues	Grower information; purchasing price; drying, impurity removal, storage, and other costs; selling price; processing enterprise information
	Dry		Drying method; moisture content before drying; moisture content after drying	Real-time ambient temperature; real-time ambient humidity		
	Impurity removal		Impurity content; impurity removal rate			
	Storage		Inventory number; product source; warehousing time; delivery time	Ambient temperature, humidity, oxygen concentration, carbon dioxide concentration, and various toxic gas concentrations produced by long-term storage		
Machining	Removing the husk	Enterprise name; business address; corporate information; person in charge of relevant links; license information; enterprise contact information	Ridge and valley mode (brand of ridge and valley machine); roughness; shelling rate	Real-time ambient temperature; real-time ambient humidity	Mycotoxin: broken needle foreign body; chemical reagents; heavy metals	Processing cost; processing price
	Rice milling		Rice milling method (chemical method/mechanical method); whole meter rate; broken rice rate			
	Color selection		Color separation accuracy; bringing out the ratio			
	Polishing		Polishing rate			
	Packing		Product package number; product batch number; product quality information			
Storage		Name of warehousing enterprise; address of storage enterprise; corporate information	Inventory number; product source; warehousing time; delivery time	Ambient temperature, humidity, oxygen concentration, carbon dioxide concentration, and various toxic gas concentrations produced by long-term storage	Mycotoxin	Storage cost; storage price
Transport		Name of logistics enterprise; address of logistics company; information of the person in charge of transportation	Means of transport; place of departure; departure time; destination	Ambient temperature inside the vehicle; ambient humidity in the vehicle; oxygen/carbon dioxide concentration in the vehicle	Fungi and toxins produced by temperature and humidity metamorphosis	Logistics cost; logistics price
Sale		Merchant name; shop address; information of the person in charge of the store; business license information; business contact information	Product name; product quantity; purchase time; purchase number; shipping time	Sales environment photos	None	Purchasing price; selling price

**Table 2:** Division mode of nodes.

Node name	Node classification	Node function
Common node	Node that reaches credit score *η* within time *t*	Can only participate in consensus
Supervision node	2(2*f* + 1)/3 nodes that first reach credit score *λ* among ordinary nodes	Can participate in consensus and can record the information of the problem node
Candidate node	2(2*f* + 1)/9 nodes that first reach credit score *μ* among ordinary nodes	Can participate in consensus and select the master node from it
Fault node	Nodes that do not reach *η* score within time *t*	Cannot participate in consensus

## Data Availability

The data supporting this study are available within the paper.
